RETRACTED

# Contamination of Hospital Water Supplies in Gilan, Iran, with *Legionella pneumophila, Escherichia coli,* and *Pseudomonas aeruginosa*

**DOI:** 10.1155/2015/809842

**Published:** 2015-09-07

**Authors:** Masoumeh Ahmadi Jalali Moghadam, Hamidreza Honarmand, Sajad Asfaram Meshginshahr

**Affiliations:** ^1^Cellular and Molecular Research Center, Guilan University of Medical Sciences, Rasht, Iran; ^2^Department of Microbiology, Guilan University of Medical Sciences, Rasht, Iran; ^3^Department of Microbiology, Islamic Azad University, Lahijan Branch, Lahijan, Iran

## Abstract

This study is designed to determine the contamination degree of hospital water supplies with *Pseudomonas aeruginosa, Legionella pneumophila*, and *E. coli* in Gilan, Iran. Samples were collected directly into sterile containers and concentrated by centrifuge. Half part of any sample transferred to yeast extract broth and the second part transferred to Trypticase Soy Broth and incubated for 3 days. DNA was extracted by using commercial kit. Four rounds of PCR were performed as follows: multiplex PCR for detecting *Pseudomonas aeruginosa*, Integron 1, and Metallo-*β*-lactamases gene; PCR for detecting *Legionella pneumophila* and *mip* gene separately; PCR for detecting *E. coli*; and another PCR for detecting whole bacterial presence. Contamination rates of cold, warm, and incubator water samples with *P. aeruginosa*, were 16.6%, 37.5%, and 6.8% consequently. Degrees of contamination with *L. pneumophila* were 3.3%, 9.3%, and 10.9% and with *E. coli* were zero, 6.2%, and zero. Total bacterial contamination of cold, warm, and incubator water samples was 93.3%, 84.4%, and 89.0% consequently. Metallo-*β*-lactamases gene was found in 20.0% of all samples. Contamination degree with *P. aeruginosa* was considerable and with *L. pneumophila* was moderate. Metallo-*β*-lactamases gene was found frequently indicating widespread multiple drug resistance bacteria. We suggest using new decontamination method based on nanotechnology.

## 1. Introduction

Nosocomial infection is an infection whose development is favored by a hospital environment. Microorganisms can be transmitted to the host by contaminated items, such as water. Water may be contaminated in many ways. The different forms of contamination come from different sources and are dealt with in different ways [1]. The three main forms of water contamination are physical, bacterial, and chemical [2]. Contamination can occur at the source, between source and storage points or in storage tanks. Defective joints, syphonage, rusted pipelines, and crossing over of sewage pipelines are other causes of contamination [3]. So, drinking water distribution systems may contain a diverse microbiological community that may include opportunistic pathogens and it is the most important single source of human exposure to gastroenteric diseases, mainly as a result of the ingestion of microbial contaminated water [4].

RETRACTED

Hospital outbreaks are usually associated with contamination of water sources [5]. Water contamination of respirators and incubators of newborns are the main sources of transfer [6, 7]. The cooling tower and the air condition system have also been reported to be sources of several outbreaks [8]. Man-made water systems especially hot water systems are main sources of* Legionella* [9]. These bacteria survive in biofilm and resist against chlorine and other disinfectants [9].

A wide variety of opportunistic pathogens such as* Pseudomonas* can be incorporated into the piped potable water, colonizing the surfaces of pipelines with high numbers of biofilm-forming bacteria [10]. In addition, in bacteriological assessments, particularly for coliforms, the indicators of contamination by fecal matter must be routinely performed by many public health authorities to ascertain the quality of water to ensure prevention of further dissemination of pathogens through the agency of water [11].

Addition of chlorine in different water treatment plants is a common practice, but it is not sufficient to ensure the safety of water. There is adverse association between bacterial count of water samples and free residual chlorine but the failure of conventional treatment processes to eliminate critical waterborne pathogens in drinking water demands that improved and/or new disinfection technologies should be developed [4].

The aim of the present study was to determine the contamination rate of cold and warm water as well as water of containers of newborn incubators in hospitals of Gilan Province, Iran, by* Pseudomonas aeruginosa, Legionella pneumophila, *and* E. coli,* using molecular approach.

## 2. Materials and Methods

### 2.1. Sampling, Processing, and Enrichment

During April–June 2014, one hundred and thirty-five water samples (about 50 mL for each) were aseptically collected in 60 mL plastic containers from 30 hospitals of the area (30 cold water samples, 32 warm water samples, and 73 incubator water samples). Cold water and warm water samples were taken after the water had run for 5 min. Water samples of incubator of newborn wards were taken directly into sterile plastic containers. Potable water is supplied to the hospitals by the municipal system where it receives no additional treatment. The water has detectable free residual chlorine upon arrival at hospitals. All water samples were concentrated 20-fold (by dividing any sample into 5 falcon tubes, centrifugation with 12000 rpm for 30 min in 4°C, discarding supernatant, dissolving precipitant in 0.5 mL remaining water, and collecting them in a tube). After discarding supernatant, sediment was resolved in 1 mL of the remaining solution and was divided into two different parts. One part was treated in 50°C for 30 min to reduce other contaminants for effective recovering of* Legionella*. After heat treatment, each sample was inoculated in 5 mL liquid medium containing yeast extract 10 g/L, L-cysteine 0.04%, ferric pyrophosphate 0.25 g/L, glycine 0.3%, and vancomycin 5 *µ*g/mL with final pH 6.9 and incubated in 35°C for 3 days. It should be noted that vancomycin and glycine are added to the medium after autoclave and when the temperature was around 40°C. The selectivity of the medium was subsequently improved by the incorporation of vancomycin and glycine. This selective medium should facilitate the recovery of Legionellaceae from environmental sources [9]. The second part of each sample was inoculated in Trypticase Soy Bean Broth and incubated in 35°C for 3 days for recovering* P. aeruginosa* and* E. coli*.

RETRACTED

### 2.2. DNA Extraction and Primers

All cultured samples were divided over 1 mL in volume and centrifuged in a Sigma model 3k30 centrifuge at 12.000 rpm in 4°C for 20 min. The supernatant was discarded, and the pellet was suspended with 1 mL of TE buffer before DNA extraction. DNA was extracted by using commercial procedure (Genomic DNA Purification Kit, Thermo Scientific, Lot: 00155557, Fermentas, Lithuania). The extracted DNA was either used immediately for PCR or stored at −20°C until analysis.

Several rounds of PCR were performed to detect* P. aeruginosa*, Integron 1, Metallo-*β*-lactamases gene,* Legionella pneumophila*,* mip* gene, and* E. coli* as the following procedure: (1) conventional PCR by using specific primers for* L. pneumophila *and* mip* gene separately, (2) multiplex PCR by using specific primers for* P. aeruginosa*, Integron 1, and Metallo-*β*-lactamases gene, (3) conventional PCR for detecting* E. coli* using specific primers, and (4) final round of PCR to investigate total presence of bacteria by using universal primers. Primers which were used in this study are characterised in Table 1.

We used genomic DNA of* L. pneumophila* type strain NCTC 11192 as positive control for the first round of PCR. A standard strain of* P. aeruginosa* (ATCC 27853) was used as positive control for the second round of PCR, and* E. coli* (ATCC 44338) was used as positive control for third and fourth rounds of PCR. Pure water was used as negative control for all rounds of PCR.

### 2.3. PCR Conditions

Two microliters of the extracted template DNA was used in a 20 *µ*L reaction mixture that included 10 *µ*L of PCR premix [Prime Taq Premix (2x), Chorea Lot number 201208], 0.5 *µ*L of each primer, and 7 *µ*L of ddH2O. Cycling program for first round amplification of* L. pneumophila *(species specific fragment) was as follows: an initial denaturation at 94°C for 5 min and then 35 cycles consisting of 94°C for 60 s, 45°C for 50 s, and 72°C for 60 s were followed by a final extension at 72°C for 10 min. Cycling program for second round of PCR was the same but the annealing temperature was 50°C. Annealing temperature for third round of PCR was 58°C and for 16S rRNA amplification with the universal primers was 47°C with the same cycling program. Electrophoresis of amplified product was performed on agarose gel (2% w/v) by 125 volts for 45 minutes and analyzed by GelDocTransluminator system (VilberLourmat model).

RETRACTED

## 3. Results

One hundred and thirty-five water samples were aseptically collected from 30 hospitals of the area (30 cold water, 32 warm water, and 73 incubator water samples). Contamination rates of cold, warm, and incubator water samples with* P. aeruginosa* were 16.6%, 37.5%, and 6.8% consequently (Tables 2 [Table tab3]–4 and Figure 1). Degrees of contamination with* L. pneumophila *were 3.3%, 9.3%, and 10.9% (Tables 2–4 and Figure 2) and with* E. coli* were zero, 6.2%, and zero (Tables 2–4 and Figure 3). Total bacterial contamination of cold, warm, and incubator water samples was 93.3%, 84.4%, and 89.0% consequently (Tables 2–4 and Figure 4).

Metallo-*β*-lactamases gene was found in 20.0% of cold water samples, 15.6% of warm water samples, and 21.9% of incubator water samples (Tables 2–4). About 60.0% of* P. aeruginosa* in incubator samples had Metallo-*β*-lactamases gene, 42.0% of warm water samples had* P. aeruginosa* with this gene, and 10.0% of* P. aeruginosa* in cold water samples had the same gene.

About 8.3% of* P. aeruginosa *in warm water samples had Integron 1 but we did not find* P. aeruginosa* with Integron 1 in any sample of incubators and cold water. We also did not find* P. aeruginosa* with both Integron 1 and Metallo-*β*-lactamases gene in incubator and cold water samples and just 1 of 12* P. aeruginosa* of warm water sample had both Integron 1 and Metallo-*β*-lactamases gene.

About 25.0% of* L. pneumophila* in incubator samples had* mip* gene and 33.3% of warm water samples had* L. pneumophila* with* mip* gene. We did not find* L. pneumophila *with* mip* gene in cold water samples.

In total, 88.9% of all samples showed bacterial contamination as revealed by PCR with universal primers, 16.3% of all samples had* P. aeruginosa*, 8.9% had* L. pneumophila*, and 1.5% had* E. coli*. The Metallo-*β*-lactamases gene was found in 20.0% and Integrin 1 was found in 3.0% of all samples.

RETRACTED

## 4. Discussion

The ability of microbes to survive in hospital water reservoir was described more than 30 years ago, and numerous studies have confirmed hospitals water as a source of nosocomial infection [19]. The bacterial contamination level related to the tap water was a point of dispersion of bacterial species, including potentially pathogenic organisms [20]. Modes of transmission for waterborne infections include direct contact, ingestion of water, indirect contact, inhalation of aerosols dispersed from water sources, and aspiration of contaminated water [21].

Several factors could be attributed to the contamination of surface water such as the age of the distribution system, the quality of the delivered water, defective chlorination, and improper maintenance [22]. Contamination can occur at the source, between source and storage points or in storage tanks [3]. The bacterial contamination occurs because of regrowth of microorganisms in biofilms which are formed on interior surfaces of water pipes. Biological activity in biofilms is controlled by nutrient content of water, temperature, and residual chlorine [23].

Microorganisms are widely distributed in nature and their abundance and diversity may be used as indicators for suitability of water [24]. Certain types of microorganisms are characteristics of human fecal contamination [25]. In the present study we used three bacteria (*E. coli*,* P. aeruginosa*, and* L. pneumophila*) to evaluate quality of studied water supplies because river and underground waters are main sources of tap water in the area and these bacteria are main human pathogens with water sources. Actually in this study,* E. coli* was used as a representative of the enteric bacterial pathogens. We also used* L. pneumophila* as ubiquitous waterborne microorganism and* P. aeruginosa* as ubiquitous waterborne opportunistic pathogen.

*E. coli* is a type of fecal coliform bacteria commonly found in the intestines of animals and humans and the presence of it in water is a strong indication of recent sewage or animal waste contamination [26]. We did not find* E. coli* in cold water and incubator water samples and just two warm water samples showed presence of* E. coli*. In some similar studies water distribution systems of examined hospitals were totally free of Gram-negative bacteria belonging to family Enterobacteriaceae [27]. Although coliforms are known as the best index for monitoring water microbial quality, in some cases this index is not very efficient. Some believe that the excess growth of heterotrophic bacteria results in suppression of the coliforms. Therefore, it is recommended to use other bacteria as an alternative index in water microbial quality control and* Pseudomonas* can be one of these indicators [28].

RETRACTED

*P. aeruginosa* is part of a large group of free-living bacteria that are ubiquitous in the environment*. P. aeruginosa* is of major concern in hospitals, since it can cause severe secondary infections, such as pneumonia in burn victims or immunocompromised persons [29]. Its occurrence in drinking water is probably related more to its ability to colonize biofilms in plumbing fixtures (i.e., faucets and showerheads) than its presence in the distribution system or treated drinking water.* P. aeruginosa* can survive in deionized or distilled water; hence, it may be found in low nutrient or oligotrophic environments such as distilled water which is used for incubators of newborn ward [30]. In the present study contamination degree of warm water with* P. aeruginosa* was higher (37.5%) than cold water (16.6%) and incubator water (6.8%). High temperatures of water can be favorable for the growth of* P. aeruginosa* [30]. It also can be isolated even in the presence of 3.00 ppm residual free chlorine [30].

A number of laboratory-based studies have demonstrated the colonization of heterogeneous biofilms developed from tap water microorganisms by pathogens such as* E. coli* [31],* L. pneumophila* [32], and* P. aeruginosa* [33]. A number of studies showed that these bacteria are important opportunistic pathogens which can be involved in biofilm-associated contamination of domestic plumbing systems [34–37].

De Abreu et al. presented that biofilm tap water was the major environmental source of pseudomonads in the healthcare facility [20]. In the present study the frequency of* P. aeruginosa* with Metallo-*β*-lactamases was 37%. It should be noted that Metallo-*β*-lactamases producing strains have been increasingly reported worldwide and have been responsible for large outbreaks in several Asian, European, and American hospitals [38–42]. Genes encoding Metallo-*β*-lactamases are generally located within class 1 integrons, together with those encoding aminoglycoside-modifying enzymes that confer multidrug resistance. In addition, the integrons harboring Metallo-*β*-lactamases determinants are frequently located on plasmids, certainly facilitating their intra- and interspecies spread [43]. High prevalence of Metallo-*β*-lactamases producing epidemic or endemic strains is also found in other Mediterranean countries, such as Italy and Greece [44].

Presence of* L. pneumophila* is associated with biofilms in warm water plumbing systems [45]. This bacterium can also survive at lower temperatures in drinking water environments [46, 47].* L. pneumophila*, particularly strains within serogroups 1 and 6, is known as cause of both community acquired and hospital associated pneumonia [48, 49]. Transmission to humans occurs through inhalation of aerosols generated from an environmental source. Several reports have demonstrated that the major sources for Legionnaires' disease are the potable water systems of large buildings including hospitals, nursing home, and hotels [50].

RETRACTED

In a similar study, Yaslianifard et al. found considerable contamination rate of* L. pneumophila* and* P. aeruginosa* in hospital water samples in Tehran, Iran [51]. Shamabadi and Ebrahimi found low rate contamination with Gram-negative flora, moderate concentrations of* Legionella*, and potentially pathogenic nonenterobacterial species [28].

In the present study we found the degree of presence of* L. pneumophila* in cold water was lower than in warm water and incubator water. It seems that high loads of* P. aeruginosa* can mask the presence of* Legionella*, leading to an underestimation in some cases. Many authors agree that different microbe species as well as high microbial loads can play an important role in limiting or even inhibiting the growth of* Legionella* [52, 53]. In our study the total bacterial contamination of cold water samples was very high (93.3%). Actually overall pollution of hospital water systems with* Legionella* found in the present work was smaller compared to earlier studies made in Germany and Italy [54–57]. In a USA national surveillance study of 20 hospitals in 13 states, 14 hospitals were colonized with* Legionella* in the water systems in which 43% of hospitals had environmental positive rates for* Legionella* [58]. In a study in Spain on 12 hospitals, the environmental positive rates for* Legionella* were ≥30% [59].* L. pneumophila* was also found in 63% of hospital water systems in Taiwan [52].

The present study showed that care should be taken concerning cleanliness and decontamination of water supplies for pathogenic organisms. Chlorine has been widely used as disinfectant due to its low cost and effectiveness in many countries but it is not sufficient to ensure the safety of water. The maintenance of chlorine residue is needed at all points in distribution system supplied with chlorine as a disinfectant [60]. The failure of conventional treatment processes to eliminate critical waterborne pathogens in drinking water demands that improved and/or new disinfection technologies be developed. Recent research has disclosed that nanotechnology may offer solutions in this area, through the use of nanosorbents, nanocatalysts, bioactive nanoparticles, nanostructured catalytic membranes, and nanoparticle-enhanced filtration [4].

RETRACTED

## 5. Conclusion

Our study demonstrated that contamination degree of studied water samples with* P. aeruginosa* was considerable, with* L. pneumophila* was moderate, and with* E. coli* was very low. We also found frequent presence of Metallo-*β*-lactamases gene in the studied water samples indicating widespread multiple drug resistance bacteria. We suggest using new decontamination method based on new disinfection technologies.

## Figures and Tables

**Figure 1:** Results of multiplex PCR with primers specific for* P. aeruginosa* species, Integron 1, and Metallo-*β*-lactamases gene, for 13 incubator samples. Line 16 is 100–1000 bp ladder. Line 15 is positive control (*P. aeruginosa* type strain ATCC 27853). Lines 5 and 12 are positive samples for* P. aeruginosa* (720 bp specific bands). Lines 2, 5, 8, and 10 are positive samples for Metallo-*β*-lactamases gene (310 bp). All samples are negative for Integrin 1. Lines 3, 4, 6, 7, 11, 13, and 14 are negative samples and line 1 is negative control (water).

**Figure 2:** Results of PCR with* L. pneumophila*: species specific primers for 13 incubator samples. Line 1 is positive control (*L. pneumophila* type strain NCTC 11192). Lines 2 and 7 are ladders (100–1000 bp). Lines 3, 4, 5, 6, 8, 10, and 11 are positive samples. Lines 9, 12, 13, 14, and 15 are negative samples and line 16 is negative control (water).

**Figure 3:** Results of PCR with* E. coli* species specific primers for 13 incubator samples. Line 16 is 100–1000 bp ladder. Line 15 is negative control (water). Line 14 is positive control (*E. coli* type strain ATCC 44338). All samples (lines 1–13) are negative.

**Figure 4:** Results of PCR with universal primer for bacterial 16S rRNA gene for 13 incubator samples. Line 2 is positive control (*E. coli *type strain* ATCC 44338*). Lines 1 and 9 are ladders (100–1000 bp). Lines 3, 4, 5, 8, 10, 11, 12, 13, 14, and 15 are positive samples. Lines 6, 7, and 13 are negative samples, and line 16 is negative control (water).

**Table 1:** Characteristic of primers used in the present study.

Primer	Sequence (5′→3′)	Use	Reference
Lpms1F Lpms1R	CAGGGAAATGCTCTAGCACAC TCGCTTCGGACTGAATTTCT	*L. pneumophila* detection	[12]

Lmip F Lmip R	GGCCAATAGGTCCGCCAACG GGTGACTGCGGCTGTTATGG	*mip* gene detection	[13]

gyrB-F gyrB-R	CCTGACCATCCGTCGCCACAAC CGCAGCAGGATGCCGACGCC	*P. aeruginosa* detection	[14]

Vim1-1A Vim1-1B	TTATGGAGCAGCAACGATGT CAAAAGTCCCGCTCCAACGA	blaVIM detection	[15]

Int1-1A Int1-1B	TACCTCTCACTAGTGAGGGG ATGAAAACCGCCACTGCGCC	int1 detection	[16]

EPE-F EPE-R	CCCGAATTCGGCACAAGCATAAGC CCCGGATCCGTCTCGCCAGTATTCG	*E. coli* detection	[17]

16srRNA F 16srRNA R	GGATTAGATACCCTGGTAGTCC TCGTTGCGGGACTTAACCCAAC	Detection of whole bacterial load	[18]

RETRACTED

**Table 2:** Summary of amplification results for cold water samples.

*P. aeruginosa *	Metallo-*β*-lactamases gene	Integron I	Coliform	*L. pneumophila*	*mip* gene	Total bacterial contamination rate
5 (30)	6 (30)	0	0	1 (30)	0	28 (30)
16.6%	20.0%	0	0	3.3%	0	93.3%

**Table 3 tab3:** Summary of amplification results for warm water samples.

*P. aeruginosa *	Metallo-*β*-lactamases gene	Integron I	Coliform	*L. pneumophila*	*mip* gene	Total bacterial contamination rate
12 (32)	5 (32)	1 (32)	2 (32)	3 (32)	1 (32)	27 (32)
37.5%	15.6%	3.1%	6.2%	9.3%	3.1%	84.4%

**Table 4:** Summary of amplification results for incubators water samples.

*P. aeruginosa *	Metallo-*β*-lactamases gene	Integron I	Coliform	*L. pneumophila*	*mip* gene	Total bacterial contamination rate
5 (73)	16 (73)	3 (73)	0	8 (73)	2 (73)	65 (73)
6.8%	21.9%	4.1%	0	10.9%	2.7%	89.0%
